# Machine Learning Based Diabetes Classification and Prediction for Healthcare Applications

**DOI:** 10.1155/2021/9930985

**Published:** 2021-09-29

**Authors:** Umair Muneer Butt, Sukumar Letchmunan, Mubashir Ali, Fadratul Hafinaz Hassan, Anees Baqir, Hafiz Husnain Raza Sherazi

**Affiliations:** ^1^School of Computer Sciences, Universiti Sains Malaysia, Penang, Malaysia; ^2^Department of Management,Information and Production Engineering, University of Bergamo, Bergamo, Italy; ^3^Department of Environmental Sciences,Informatics,and Statistics, Ca'Foscari University of Venice, Venice, Italy; ^4^School of Computing and Engineering, University of West London, London, UK

## Abstract

The remarkable advancements in biotechnology and public healthcare infrastructures have led to a momentous production of critical and sensitive healthcare data. By applying intelligent data analysis techniques, many interesting patterns are identified for the early and onset detection and prevention of several fatal diseases. Diabetes mellitus is an extremely life-threatening disease because it contributes to other lethal diseases, i.e., heart, kidney, and nerve damage. In this paper, a machine learning based approach has been proposed for the classification, early-stage identification, and prediction of diabetes. Furthermore, it also presents an IoT-based hypothetical diabetes monitoring system for a healthy and affected person to monitor his blood glucose (BG) level. For diabetes classification, three different classifiers have been employed, i.e., random forest (RF), multilayer perceptron (MLP), and logistic regression (LR). For predictive analysis, we have employed long short-term memory (LSTM), moving averages (MA), and linear regression (LR). For experimental evaluation, a benchmark PIMA Indian Diabetes dataset is used. During the analysis, it is observed that MLP outperforms other classifiers with 86.08% of accuracy and LSTM improves the significant prediction with 87.26% accuracy of diabetes. Moreover, a comparative analysis of the proposed approach is also performed with existing state-of-the-art techniques, demonstrating the adaptability of the proposed approach in many public healthcare applications.

## 1. Introduction

Public health is a fundamental concern for protecting and preventing the community from health hazard diseases [1]. Governments are spending a considerable amount of their gross domestic product (GDP) for the welfare of the public, and initiatives such as vaccination have prolonged the life expectancy of people [2]. However, for the last many years, there has been a considerable emergence of chronic and genetic diseases affecting public health. Diabetes mellitus is one of the extremely life-threatening diseases because it contributes to other lethal diseases, i.e., heart, kidney, and nerve damage [3].

Diabetes is a metabolic disorder that impairs an individual's body to process blood glucose, known as blood sugar. This disease is characterized by hyperglycemia resulting from defects in insulin secretion, insulin action, or both [3]. An absolute deficiency of insulin secretion causes type 1 diabetes (T1D). Diabetes drastically spreads due to the patient's inability to use the produced insulin. It is called type 2 diabetes (T2D) [4]. Both types are increasing rapidly, but the ratio of increase in T2D is higher than T1D. 90 to 95% of cases of diabetes are of T2D.

Inadequate supervision of diabetes causes stroke, hypertension, and cardiovascular diseases [5]. To avoid and reduce the complications due to diabetes, a monitoring method of BG level plays a prominent role [6]. A combination of biosensors and advanced information and communication technology (ICT) provides an efficient real-time monitoring management system for the health condition of diabetic patients by using SMBG (self-monitoring of blood glucose) portable device. A patient can check the changes in glucose level in his blood by himself [7]. Users can better understand BG changes by using CGM (continuous glucose monitoring) sensors [4].

By exploiting the advantages of the advancement in modern sensor technology, IoT, and machine learning techniques, we have proposed an approach for the classification, early-stage identification, and prediction of diabetes in this paper. The primary objective of this study is twofold. First, to classify diabetes into predefined categories, we have employed three widely used classifiers, i.e., random forest, multilayer perceptron, and logistic regression. Second, for the predictive analysis of diabetes, long short-term memory (LSTM), moving averages (MA), and linear regression (LR) are used. To demonstrate the effectiveness of the proposed approach, PIMA Indian Diabetes is used for experimental evaluation. We concluded that, in experimental evaluation, MLP achieved an accuracy of 86.083% in diabetes classification as compared to the other classifiers and LSTM achieved a prediction accuracy of 87.26% for the prediction of diabetes. Moreover, we have also performed a comparative analysis of the proposed approach with existing state-of-the-art approaches. The accuracy results of our proposed approach demonstrate its adaptability in many healthcare applications.

Besides, we have also presented the IoT-based hypothetical diabetes self-monitoring system that uses BLE (Bluetooth Low Energy) devices and data processing in real-time. The latter technique used two applications: Apache Kafka (for streaming messages and data) and MongoDB (to store data). By utilizing BLE-based sensors, one can collect essential sign data about weight and blood glucose. These data will be handled by data processing techniques in a real-time environment. A BLE device will receive all the data produced by sensors and other necessary information about the patient that resides in the user application, installed on the cell phone. The raw data produced by sensors will be processed using the proposed approach to produce results, suggestions, and treatment from the patient's server-side.

The rest of the paper is organized as follows. In Section 2, the paper presents the motivations for the proposed system by reviewing state-of-the-art techniques and their shortcomings. It covers the literature review about classification, prediction, and IoT-based techniques for healthcare.  Section 3 highlights the role of physical activity in diabetes prevention and control. In Section 4, we proposed the design and architecture of the diabetes classification and prediction systems.  Section 5 discusses the results and performance of the proposed approach with state-of-the-art techniques. In Section 6, an IoT-based hypothetical system is presented for real-time monitoring of diabetes. Finally, the paper is concluded in Section 7, outlining the future research directions.

## 2. Literature Review

In this section, we discussed the classification and prediction algorithms for diabetes prediction in healthcare. Particularly, the significance of BLE-based sensors and machine learning algorithms is highlighted for self-monitoring of diabetes mellitus in healthcare. Machine learning plays an essential part in the healthcare industry by providing ease to healthcare professionals to analyze and diagnose medical data [8–12]. Moreover, intelligent healthcare systems are providing real-time clinical care to needy patients [13, 14]. The features covered in this study are compared with the state-of-the-art studies (Table 1).

### 2.1. Diabetes Classification for Healthcare

Health condition diagnosis is an essential and critical aspect for healthcare professionals. Classification of a diabetes type is one of the most complex phenomena for healthcare professionals and comprises several tests. However, analyzing multiple factors at the time of diagnosis can sometimes lead to inaccurate results. Therefore, interpretation and classification of diabetes are a very challenging task. Recent technological advances, especially machine learning techniques, are incredibly beneficial for the healthcare industry. Numerous techniques have been presented in the literature for diabetes classification.

Qawqzeh et al. [15] proposed a logistic regression model based on photoplethysmogram analysis for diabetes classification. They used 459 patients' data for training and 128 data points to test and validate the model. Their proposed system correctly classified 552 persons as nondiabetic and achieved an accuracy of 92%. However, the proposed technique is not compared with state-of-the-art techniques. Pethunachiyar [16] presented a diabetes mellitus classification system using a machine learning algorithm. Mainly, he used a support vector machine with different kernel functions and diabetes data from the UCI Machine Repository. He found SVM with linear function more efficient than naïve Bayes, decision tree, and neural networks. Nevertheless, the state-of-the-art comparison is missing and parameter selection is not elaborated.

Gupta et al. [17] exploited naïve Bayes and support vector machine algorithms for diabetes classification. They used the PIMA Indian Diabetes dataset. Besides, they used a feature selection based approach and k-fold cross-validation to improve the accuracy of the model. The experimental results showed the supremacy of the support vector machine over the naïve Bayes model. However, state-of-the-art comparison is missing along with achieved accuracy. Choubey et al. [18] presented a comparative analysis of classification techniques for diabetes classification. They used PIMA Indian data collected from the UCI Machine Learning Repository and a local diabetes dataset. They used AdaBoost, K-nearest neighbor regression, and radial basis function to classify patients as diabetic or not from both datasets. Besides, they used PCA and LDA for feature engineering, and it is concluded that both are useful with classification algorithms for improving accuracy and removing unwanted features.

Maniruzzaman et al. [19] used a machine learning paradigm to classify and predict diabetes. They utilized four machine learning algorithms, i.e., naive Bayes, decision tree, AdaBoost, and random forest, for diabetes classification. Also, they used three different partition protocols along with the 20 trials for better results. They used US-based National Health and Nutrition Survey data of diabetic and nondiabetic individuals and achieved promising results with the proposed technique. Ahuja et al. [20] performed a comparative analysis of various machine learning approaches, i.e., NB, DT, and MLP, on the PIMA dataset for diabetic classification. They found MLP superior as compared to other classifiers. The authors suggested that the performance of MLP can be enhanced by fine-tuning and efficient feature engineering. Recently, Mohapatra et al. [21] have also used MLP to classify diabetes and achieved an accuracy of 77.5% on the PIMA dataset but failed to perform state-of-the-art comparisons. MLP has been used in the literature for various healthcare disease classifications such as cardiovascular and cancer classification [35, 36].

### 2.2. Predictive Analysis of Diabetes for Healthcare

Accurate classification of diabetes is a fundamental step towards diabetes prevention and control in healthcare. However, early and onset identification of diabetes is much more beneficial in controlling diabetes. The diabetes identification process seems tedious at an early stage because a patient has to visit a physician regularly. The advancement in machine learning approaches has solved this critical and essential problem in healthcare by predicting disease. Several techniques have been proposed in the literature for diabetes prediction.

Singh and Singh [22] proposed a stacking-based ensemble method for predicting type 2 diabetes mellitus. They used a publicly available PIMA dataset from the UCI Machine Learning Repository. The stacking ensemble used four base learners, i.e., SVM, decision tree, RBF SVM, and poly SVM, and trained them with the bootstrap method through cross-validation. However, variable selection is not explicitly mentioned and state-of-the-art comparison is missing.

Kumari et al. [23] presented a soft computing-based diabetes prediction system that uses three widely used supervised machine learning algorithms in an ensemble manner. They used PIMA and breast cancer datasets for evaluation purposes. They used random forest, logistic regression, and naïve Bayes and compared their performance with state-of-the-art individual and ensemble approaches, and their system outperforms with 79% accuracy.

Islam et al. [24] utilized data mining techniques, i.e., random forest, logistic regression, and naïve Bayes algorithm, to predict diabetes at the early or onset stage. They used 10-fold cross-validation and percentage split techniques for training purposes. They collected diabetic and nondiabetic data from 529 individuals directly from a hospital in Bangladesh through questionnaires. The experimental results show that random forest outperforms as compared to other algorithms. However, the state-of-the-art comparison is missing and achieved accuracy is not reported explicitly.

Malik et al. [25] performed a comparative analysis of data mining and machine learning techniques in early and onset diabetes mellitus prediction in women. They exploited traditional machine learning algorithms for proposing a diabetes prediction framework. The proposed system is evaluated on a diabetes dataset of a hospital in Germany. The empirical results show the superiority of K-nearest neighbor, random forest, and decision tree compared to other traditional algorithms.

Hussain and Naaz [26] presented a thorough review of machine learning models presented during 2010–2019 for diabetes prediction. They compared traditional supervised machine learning models with neural network-based algorithms in terms of accuracy and efficiency. They used Matthews correlation coefficient for evaluation purposes and observed naïve Bayes and random forest's supremacy compared to other algorithms.

### 2.3. Real-Time IoT-Based Processing of Healthcare Data

Real-time diabetes prediction is a complicated task. The emerging use of sensors in healthcare paved the path to handle fatal diseases [37]. Several techniques have been presented in the literature to classify and predict diabetes. Acciaroli et al. [4] exposed two accurate meters to measure diabetes in blood with less error rate. Furthermore, these commercial versions of glucometers are Accu-Chek with 6.5% error and CareSens with 4.0% error. Buckingham et al. [38] described the accuracy link of CGM with the calibration sensor. Alfian et al. [27] uncovered that the FDA had accepted CGM sensors for monitoring glucose in different trends and patterns. Moreover, at one particular time, one glucose reading should not be used to analyze the amount of insulin as not accepted in a glucometer. Rodríguez et al. [28] proposed a structural design containing a local gateway as a smartphone, cloud system, and sensors for advanced management of diabetes.

Filippoupolitis et al. [29] planned action to acknowledge a system using Bluetooth Low Energy (BLE) beacons and smartwatches. Mokhtari et al. considered technologies working with BLE for activity labeling and resident localization [30]. Gentili et al. [31] have used BLE with another application called Blue Voice, which can reveal the probability of multimedia communication of sensor devices and speech streaming service. Suárez et al. [32] projected a monitoring system based on the BLE device for air quality exposure with the environmental application. It aims at defining potential policy responses and studies the variables that are interrelated between societal level factors and diabetes prevalence [33, 34].

Wang et al. [39] have given a general idea of the up-to-date BLE technology for healthcare systems based on a wearable sensor. They suggested that low-powered communication sensor technologies such as a BLE device can make it feasible for wearable systems of healthcare because it can be used without location constraints and is light in weight. Moreover, BLE is the first wireless technology in communication for healthcare devices in the form of a wearable device that meets expected operating requirements with low power, communication with cellular directly, secure data transmission, interoperability, electronic compatibility, and Internet communications. Rachim and Chung [40] have suggested one transmission system that used deficient power to observe the heart's activity through electrocardiograph signals using a BLE device for data transmission collecting by armband sensors and smartphones.

Mora et al. projected a dispersed structure using the IoT model to check human biomedically generated signals in reports using a BLE sensor device [41]. Cappon et al. [42] explored the study of CGM wearable sensors' prototypes and features of the commercial version currently used. Årsand et al. [43] offered the easiest method for monitoring blood glucose, physical activity, insulin injections, and nutritional information using smartphones and smartwatches. Morón et al. [44] observed the performance of the smartphone used in the medical field. Lee and Yoo [45] anticipated a structure using PDA (personal digital assistant) to manage diabetic patient's conditions better. It can also be used to send information about blood pressure, BG level, food consumption, and exercise plan of a patient with diabetes and give the direction of treatment by monitoring physical activity, food consumption, and insulin prescribed amount.

Rodríguez et al. [28] suggested an application for the smartphone, which can be used to receive the data from the sensor using a glucometer automatically. Rodríguez-Rodríguez et al. [46] suggested that checking the patient's glucose level and heart rate using sensors will produce colossal data, and analysis on big data can be used to solve this problem.

## 3. Role of Physical Activity in Prevention and Control of Diabetes Mellitus

Generally, physical activity is the first prevention and control strategy suggested by healthcare professionals to diabetic or prediabetic patients [47]. Among diet and medicine, exercise is a fundamental component in diabetes, cardiovascular disease, obesity, and lifestyle rescue programs. Nonetheless, dealing with all the fatal diseases has a significant economic burden. However, diabetes mellitus emerged as a devastating problem for the health sector and economy of a country of this century.

Recently, the international diabetes prevention and control federation predicts that diabetes can affect more than 366 million people worldwide [49]. The disease control and prevention center in the US alarmed the government that diabetes can affect more than 29 million people [50]. While these alarming numbers are continuously increasing, they will burden the economy around the globe. Therefore, researchers and healthcare professionals worldwide are researching and proposing guidelines to prevent and control this life-threatening disease. Sato [51] presented a thorough survey on the importance of exercise prescription for diabetes patients in Japan. He suggested that prolonged sitting should be avoided and physical activity should be performed every 30 minutes. Kirwan et al. [47] emphasized regular exercise to control and prevent type 2 diabetes. Particularly, they studied the metabolic effect on tissues of diabetic patients and found very significant improvements in individuals performing regular exercise. Moser et al. [48] have also highlighted the significance of regular exercise in improving the functionality of various organs of the body, as shown in Figure 1.

Yang et al. [52] focused on exercise therapy which plays a significant role in treating diabetes and its associated side effects. Specifically, they discovered cytokines which gives a novel insight into diabetes control, but the sequence is still under study. Kim and Jeon [53] presented a systematic overview of the effect of different exercises on the metabolism improvement of diabetic young individuals. They pointed out that several studies reported the significance of exercise on insulin, BP, and BG level improvement. However, none of these studies mentions the beta-cell improvement. Therefore, many challenges persist in diabetes prevention and control, which need serious attention from researchers worldwide.

## 4. Proposed Diabetic Classification and Prediction System for Healthcare

The proposed diabetes classification and prediction system has exploited different machine learning algorithms. First, to classify diabetes, we utilized logistic regression, random forest, and MLP. Notably, we fine-tuned MLP for classification due to its promising performance in healthcare, specifically in diabetes prediction [20, 21, 35, 36]. The proposed MLP architecture and algorithm are shown in Figure 2 and Algorithm 1, respectively.

Second, we implement three widely used machine learning algorithms for diabetes prediction, i.e., moving averages, linear regression, and LSTM. Mainly, we optimized LSTM for crime prediction due to its outstanding performance in real-world applications, particularly in healthcare [53]. The implementation details of the proposed algorithms are as follows.

### 4.1. Diabetes Classification Techniques

For diabetic classification, we fine-tuned three widely used state-of-the-art techniques. Mainly, a comparative analysis is performed among the proposed techniques for classifying an individual in either of the diabetes categories. The details of the proposed diabetes techniques are as follows.

#### 4.1.1. Logistic Regression

It is appropriate to use logistic regression when the dependent variable is binary [54], as we have to classify an individual in either type 1 or type 2 diabetes. Besides, it is used for predictive analysis and explains the relationship between a dependent variable and one or many independent variables, as shown in equation (1). Therefore, we used the sigmoid cost function as a hypothesis function (*h*_*θ*_(*x*)). The aim is to minimize cost function *J*(*θ*). It always results in classifying an example either in class 1 or class 2.

(1) $$\begin{array}{c} h_{\theta }\left(x\right)=\frac{1}{1+e^{-\theta^{T}x}},\\ J\left(\theta \right)=-\frac{1}{m}\left[\overset{m}{\underset{i=1}{\sum }}y^{i}\log\;h_{\theta }\left(x^{i}\right)+\left(1-y^{i}\right)\text{ log}\left(1-h_{\theta }\left(x^{i}\right)\right)\right]. \end{array}$$

#### 4.1.2. Random Forest (RF)

As its name implies, it is a collection of models that operate as an ensemble. The critical idea behind RF is the wisdom of the crowd, each model predicts a result, and in the end, the majority wins. It has been used in the literature for diabetic prediction and was found to be effective [55]. Given a set of training examples *X* = *x*_1_, *x*_2_,…, *x*_*m*_ and their respective targets *Y* = *y*_1_, *y*_2_,…, *y*_*m*_, RF classifier iterates B times by choosing samples with replacement by fitting a tree to the training examples. The training algorithm consists of the following steps depicted in equation (2).

- For *b* = 1...*B*, sample with replacement *n* training examples from *X* and *Y*.
- Train a classification tree *f*_*b*_ on *X*_*b*_ and *Y*_*b*_.

(2) $$\begin{array}{c} f=\frac{1}{B}\overset{B}{\underset{b=1}{\sum }}f_{b}\left(x{}^{\prime }\right). \end{array}$$

#### 4.1.3. Multilayer Perceptron

For diabetes classification, we have fine-tuned multilayer perceptron in our experimental setup. It is a network where multiple layers are joined together to make a classification method, as shown in Figure 2. The building block of this model is perceptron, which is a linear combination of input and weights. We used a sigmoid unit as an activation function shown in Algorithm 1. The proposed algorithm consists of three main steps. First, weights are initialized and output is computed at the output layer (*δ*_*k*_) using the sigmoid activation function. Second, the error is computed at hidden layers (*δ*_*h*_) for all hidden units. Finally, in a backward manner, all network weights (*w*_*i*,*j*_) are updated to reduce the network error. The detailed procedure is outlined in Algorithm 1 for diabetes classification.

Figure 2 shows the multilayer perceptron classification model architecture where eight neurons are used in the input layer because we have eight different variables. The middle layer is the hidden layer where weights and input will be computed using a sigmoid unit. In the end, results will be computed at the output layer. Backpropagation is used for updating weights so that errors can be minimized for predicting class labels. For simplicity, only one hidden layer is shown in the architecture, which in reality is much denser.

Input data from the input layer are computed on the hidden layers with the input values and weights initialized. Every unit in the middle layer called the hidden layer takes the net input, applies activation function “sigmoid” on it, and transforms the massive data into a smaller range between 0 and 1. The calculation is functional for every middle layer. The same procedure is applied on the output layer, which leads to the results towards the prediction for diabetes.

### 4.2. Diabetes Prediction

It is more beneficial to identify the early symptoms of diabetes than to cure it after being diagnosed. Therefore, in this study, a diabetes prediction system is proposed where three state-of-the-art machine learning algorithms are exploited, and a comparative analysis is performed. The details of the proposed approaches are as follows.

#### 4.2.1. Moving Averages

To predict diabetes, we used moving averages with the experimental setup due to its effectiveness in diabetes prediction for children [56]. It is based on a calculation that analyzes data points by creating a series of averages of the subset of the data randomly. The moving average algorithm is based on the “forward shifting” mechanism. It excludes the first number from the series and includes the next value in the dataset, as shown in equation (3). The input values are calculated by averaging (*P*_*SM*_) the train data at certain time stamps *P*_*M*_ + *P*_*M*_ + … P_*M*−(*n*−1)_. The algorithm used past observations as input and predicted future events.

(3) $$\begin{array}{c} P_{SM}=\frac{P_{M}+\;P_{M-1}+\ldots +P_{M-\left(n-1\right)}}{n}\\ =\frac{1}{n}\overset{n-1}{\underset{i=0}{\sum }}P^{M-i}. \end{array}$$

#### 4.2.2. Linear Regression

Second, a linear regression model is applied to the PIMA Indian dataset with the same experimental setup. We used this approach to model a relationship between a dependent variable, that is, outcome in our case, and one or more independent variables. The autonomous variable response affects a lot on the target/dependent variable, as shown in equation (4). We use a simplified hypothesis and cost function for multivariate linear regression, as there are eight different variables in our dataset [57]. We choose a very simplified hypothesis function (*h*_*θ*_(*x*)). The aim is to minimize cost function *J*(*θ*) by choosing the suitable weight (*θ*^*T*^*x*) parameters and minimizing sum of squared error (SSE).

(4) $$\begin{array}{c} J\left(\theta \right)=\frac{1}{2m}\overset{m}{\underset{i=1}{\sum }}{\left(h_{\theta }\left(x^{\left(i\right)}-y^{i}\right)\right)}^{2}\\ h_{\theta }\left(x\right)=\theta^{T}x\\ =\theta_{0}x_{0}+\theta_{1}x_{1}+\cdots +\theta_{n}x_{n}. \end{array}$$

#### 4.2.3. Long Short-Term Memory

For diabetic forecasting, we have calibrated the long short-term memory algorithm with our experimental setup. The proposed approach outperformed as compared to other state-of-the-art techniques implemented, as shown in Table 2. LSTM is based on recurrent neural network (RNN) architecture, and it has feedback connections that make it suitable for diabetes forecasting [58]. LSTM mainly consists of a cell, keep gate, write gate, and an output gate, as shown in Figure 3. The key behind using LSTM for this problem is that the cell remembers the patterns over a long period, and three portals help regulate the information flow in and out of the system. The details are presented in Algorithm 2.

Input to the algorithm is eight attributes enlisted in Table 3, measured from healthy and diabetic patients. The proposed LSTM-based diabetes prediction algorithm is trained with 80% of the data, and the remaining 20% is used for testing. We fine-tuned the prediction model by using a different number of LSTM units in the cell state. This fine-tuning helps to identify more prominent features in the dataset. These features will be kept in the cell state of the keep gate of the LSTM and will be given more weightage because they provide more insights to predict BG level. After that, we updated the network's weights by pointwise addition of the cell state and passed only those essential attributes for BG prediction. At this stage, we captured the dependencies between diabetes parameters and the output variable. Finally, the output gate updates the cell state and outputs/forwards only those variables that can be mapped efficiently on the outcome variable.

The diabetes prediction algorithm consists of three fundamental steps. First, weights are initialized and a sigmoid unit is used in the forget/keep gate to decide which information should be retained from previous and current inputs (*C*_*t*−1_, *h*_*t*−1_,  and *x*_*t*_). The input/write gate takes the necessary information from the keep gate and uses a sigmoid unit which outputs a value between 0 and 1. Besides, a Tan_h_ unit is used to update the cell state *C*_*t*_ and combine both outputs to update the old cell state to the new cell state.

Finally, inputs are processed at the output gate and again a sigmoid unit is applied to decide which cell state should be output. Also, Tan_h_ is applied to the incoming cell state to push the output between 1 and −1. If the output of the gate is 1, then the memory cell is still relevant to the required production and should be kept for future results. If the output of the gate is 0, the memory cell is not appropriate, so it should be erased. For the write gate, the suitable pattern and type of information will be determined written into the memory cell. The proposed LSTM model predicts the BG level (*h*_*t*_) as output based on the patient's existing BG level (*X*_*t*_).

## 5. Experimental Studies

The proposed diabetes classification and prediction algorithm is evaluated on a publicly available PIMA Indian Diabetes dataset (https://www.niddk.nih.gov/health-information/diabetes). Besides, a comparative analysis is performed with state-of-the-art algorithms. The experimental results show the supremacy of the proposed algorithm as compared to state-of-the-art algorithms. The details of the dataset, performance measures, and comparative analysis performed are described in the following sections.

### 5.1. Dataset

This study used the PIMA Indian Diabetes (PID) dataset taken from the National Institute of Diabetes and Kidney Diseases center [59]. The primary objective of using this dataset is to build an intelligent model that can predict whether a person has diabetes or not, using some measurements included in the dataset. There are eight medical predictor variables and one target variable in the dataset. Diabetes classification and prediction are a binary classification problem. The details of the variables are shown in Table 3.

The dataset consists of 768 records of different healthy and diabetic female patients of age greater than twenty-one, as shown in Figure 4. The feature value distribution is shown in Figure 5. The target variable outcome contains only two values, 0 and 1. The primary objective of using this dataset was to predict diabetes diagnostically. Whether a user has a chance of diabetes in the coming four years in women belongs to PIMA Indian. The dataset has a total of eight variables: glucose tolerance, no. of pregnancies, body mass index, blood pressure, age, insulin, and Diabetes Pedigree Function. All eight attributes shown in Table 3 are used for the training dataset in the classification model in this work.

### 5.2. Experimental Result and Discussion

This paper compares the proposed diabetes classification and prediction system with state-of-the-art techniques using the same experimental setup on the PIMA Indian dataset. The following sections highlighted the performance measure used and results attained for classification and prediction, and a comparative analysis with baseline studies is presented.

#### 5.2.1. Performance Metrics

Three widely used state-of-the-art performance measures (Recall, Precision, and Accuracy) are used to evaluate the performance of proposed techniques, as shown in Table 4. TP shows a person does not have diabetes and identified as a nondiabetic patient, and TN shows a diabetic patient correctly identified as a diabetic patient. FN shows the patient has diabetes but is predicted as a healthy person. Moreover, FP shows the patient is a healthy person but predicted as a diabetic patient. The algorithm utilized 10-fold cross-validation for training and testing the classification and prediction model.

For diabetes prediction, the two most commonly used performance measures are the means correlation coefficient (*r*/Pearson *R*) and root mean square error (RMSE), as shown in Table 5. *R* is mainly used to measure the linear dependence strength among the two variables. One variable is for actual value, and another variable is for predicted values. RMSE generates a hint of the overall correctness of the estimate. There can be three values for correlation: 0 for no relation, 1 for positive correlation, and −1 for the negative correlation. RMSE shows the difference between actual values and predicted values.

#### 5.2.2. Attained Results of Diabetic Classification Technique

For diabetic classification, three state-of-the-art classifiers are evaluated on the PIMA dataset. The results illustrate that the fine-tuned MLP algorithm obtained the highest accuracy of 86.083% as compared to state-of-the-art systems, as shown in Table 2.

It is evident from the results that our proposed calibrated MLP model could be used for the effective classification of diabetes. The proposed classification approach can also be beneficial in the future with our proposed hypothetical system. Data of weight scales, blood pressure monitor, and blood glucometer will be collected through sensor devices such as BLE and input of user's demographic data (for example, date of birth, height, and age). The proposed MLP algorithm outperforms with 86.6% Precision, 85.1% Recall, and 86.083% Accuracy, as shown in Figure 6. These results are outstanding for decision-making with the proposed hypothetical system to determine patient diabetes, T1D or T2D.

We also have explored the dataset used in Andy Choens' study [27]. This dataset consists of records of only one patient. The information was recorded every five minutes. The collection of data was made by using a sensor device (a CGM device). This device allows the patient to store information about BG every five minutes. So, the recorded data by using this device are in massive amounts. Dataset was limited, and most data were noisy that can affect the accuracy of the proposed system, so we neglected it.

#### 5.2.3. Achieved Results of Diabetic Prediction Techniques

For diabetic prediction, we implemented three state-of-the-art algorithms, i.e., linear regression, moving averages, and LSTM. Notably, we fine-tuned LSTM and compared its performance with other algorithms. It is evident from Figure 7 and Table 6 that the LSTM outperformed as compared to other algorithms implemented in this study.

Table 2 shows the performance values of prediction models with RMSE and *r* evaluation measures. The proposed fine-tuned LSTM produced the highest accuracy, 87.26%, compared to linear regression and moving average. We can see in Table 6 that the correlation coefficient value is 0.999 using LSTM, −0.071 for linear regression, and 0.710 for moving average, as shown in Figure 7.

#### 5.2.4. Comparison of the Proposed Method with Baseline Studies

Different baseline studies have been implemented and compared with the proposed system to verify the performance of the proposed diabetes classification and prediction system. Mainly, we focus on those studies that used the PIMA dataset.

First, we compare the state-of-the-art diabetes classification techniques with the proposed technique. All the baseline techniques [17–19] used the PIMA dataset and the same evaluation measures used in this study. In particular, the authors compared naïve Bayes [17], PCA_CVR (classification via regression) [18], and SVM [19] with different machine learning techniques for diabetes classification. However, the proposed fine-tuned MLP-based diabetes classification technique outperformed as compared to baseline studies, as shown in Figure 8.

Several attempts have also been made in the literature for diabetic prediction due to its importance in real life. For this comparison, we have chosen the most recent and state-of-the-art techniques. We compare the proposed system performance with the recent state-of-the-art systems [60–65], as shown in Figure 9 and Table 7. The proposed method outperformed as compared to state-of-the-art systems with an accuracy of 87.26%, all the compared systems evaluated on the PID with the same experimental setup.

## 6. Proposed Hypothetical IoT-Based Diabetic Monitoring System for Healthcare

This study has also proposed the architecture of a hypothetical diabetic monitoring system for diabetic patients. The proposed hypothetical system will enable a patient to control, monitor, and manage their chronic conditions in a better way at their homes. The monitoring system will store the health activities and create interaction between patients, smartphones, sensor medical devices, web servers, and medical teams by providing a platform having wireless communication devices, as shown in Figure 10. The central theme of the proposed healthcare monitoring system is the collection of data from sensors using wireless devices and transmitting to a remote server for diagnosis and treatment of diabetes. Knowledge-based data are stored. Rule-based procedures will be applied for the suggestions and treatment of diabetes, informing the patient about his current health condition, prediction, and recommendation of future changes in BG.

First, essential data about patient health will be collected from sensors such as BLE wireless devices. Data comprised weight, blood pressure, blood glucose, and heartbeat, along with some demographic information such as age, sex, name, and CNIC (Social Security Number). Some information is required in the application installed on the user's mobile and sensor data. All completed data in the application will be transferred to the real-time data processing system. On the other side, aggregate data will be stored in MongoDB for future processing. Analysis and prepossessing techniques are performed to extract rules from the knowledge base for the treatment and suggestions about the user. Results and treatment procedures will be sent to the monitoring system, and finally, the user can get the output by interacting with their android mobile phone. In the end, the patient will know about the health condition and risk prediction of diabetes based on the data transferred by their application and stored data from history about the user.

### 6.1. Tools and Technology for Implementation of Hypothetical System for Healthcare

The proposed structural design for hypothetical real-time processing and monitoring of diabetes is shown in Figure 11. The data from the user's mobile will be transmitted in the JavaScript Object Notation (JSON) format to the Application Program Interface (API) in any language. The data produced at this stage will be in the form of messages, which are then transferred to the Kafka application [27]. Kafka will store all the data and messages and deliver the required data and processed output to the endpoints that could be a web server, monitoring system, or a database for permanent storage. In Kafka, application data are stored in different brokers, which can cause latency issues. Therefore, within the system architecture, it is vital to consider processing the readings from the sensors closer to the place where data are acquired, e.g., on the smartphone. The latency problem could be solved by placing sensors close to the place, such as a smartphone where data are sent and received.

This inclusion will make the overall network architecture compliant to the emerging Edge and Fog computing paradigms, whose importance in critical infrastructures such as hospitals is gaining momentum. It is essential to consider the Edge and Fog computation paradigm while sending and receiving data from smartphones to increase the performance of the hypothetical system. Edge computing utilizes sensors and mobile devices to process, compute, and store data locally rather than cloud computing. Besides, Fog computing places resources near data sources such as gateways to improve latency problems [9].

Apache Kafka will be used in real time as a delivery agent for messages in a platform that allows fault-tolerant, tall throughput, and low-latency publication. The vital signs' data collected by the patients are placed using the JSON format and then transmitted using wireless devices with the help of an android application having HTTP along with REST API for the confined remote server for the design [28]. Moreover, Node.js for web design will be used as a REST API to collect sensor data. Kafka application will receive it in the form of streams of records.

The sensor data that comes from the Kafka application is continuously generated and stored on the server. In the proposed system, the MongoDB NoSQL database will be used for data storage due to its efficiency in handling and processing real-world data [29]. The stored diabetes patient data can be input into our proposed diabetes classification and prediction techniques to get useful insights.

## 7. Conclusion

In this paper, we have discussed an approach to assist the healthcare domain. The primary objective of this study is twofold. First, we proposed an MLP-based algorithm for diabetes classification and deep learning based LSTM for diabetes prediction. Second, we proposed an IOT-based hypothetical real-time diabetic monitoring system. The proposed theoretical diabetic monitoring system will use a smartphone, BLE-based sensor device, and machine learning based methods in the real-time data processing environment to predict BG levels and diabetes. The primary objective of the proposed system is to help the users monitor their vital signs using BLE-based sensor devices with the help of their smartphones.

Moreover, the proposed model will help the users to find out the risk of diabetes at a very early stage and help them gaining future predictions of their BG increase levels. For diabetic classification and prediction, MLP and LSTM are fine-tuned. The proposed approaches are evaluated on the PIMA Indian Diabetes dataset. Both approaches are compared with state-of-the-art approaches and outperformed with an accuracy of 86.083% and 87.26%, respectively.

As future work, we plan to implement the android application for the proposed hypothetical diabetic monitoring system with the proposed classification and prediction approaches. Genetic algorithms can also be explored with the proposed prediction mechanism for better monitoring [24, 64, 66–71].

## Figures and Tables

**Figure 1:** Impact of regular exercise on metabolism of diabetic patients [48].

**Figure 2:** Proposed MLP architecture with eight variables as input for diabetes classification.

**Figure 3:** BG prediction using long short-term memory (LSTM) algorithm.

**Figure 4:** PIMA data distribution.

**Figure 5:** Dataset features' distribution visualization.

**Figure 6:** Performance comparison of classifiers.

**Figure 7:** Performance comparison of forecasting model.

**Figure 8:** Proposed diabetes classification method vs. state-of-the-art techniques.

**Figure 9:** Proposed diabetes prediction method vs. state-of-the-art systems.

**Figure 10:** The proposed hypothetical architecture of the healthcare monitoring system.

**Figure 11:** Implementation level details of the proposed hypothetical system.

**Algorithm 1:** Diabetes classification algorithm using MLP for healthcare.

**Algorithm 2:** Diabetes prediction algorithm by exploiting LSTM for healthcare.

**Table 1:** Features' comparison of the proposed study vs. state-of-the-art studies.

Study	Diabetes classification	Diabetes prediction	Real-time healthcare data analysis	Performance measures
[15]	✔	✖	✖	Accuracy
[16]	✔	✖	✖	NA
[17]	✔	✖	✖	Accuracy
[18]	✔	✖	✖	NA
[19]	✔	✔	✖	Accuracy
[20]	✔	✖	✖	Accuracy
[21]	✔	✖	✖	NA
[22]	✖	✔	✖	Accuracy
[23]	✔	✔	✖	Accuracy
[24]	✖	✔	✖	Accuracy
[25]	✖	✔	✖	Accuracy
[26]	✖	✔	✖	Accuracy, correlation coefficient
[4]	✖	✖	✔	NA
[27–33]	✖	✖	✔	NA
[34]	✔	✖	✔	Accuracy
[8]	✔	✖	✔	Accuracy, standard deviation
Proposed	✔	✔	✔	Accuracy, Precision, Recall, RMSE, *r*

**Table 2:** Performance comparison of classifiers in diabetes classification.

Algorithm	Accuracy (%)	Recall (%)	Precision (%)
Logistic regression	73.05	72.7	73
Random forest	77.4	75.7	76.9
Proposed fine-tuned MLP	86.083	85.1	86.6

**Table 3:** Description of variables in the dataset.

Attributes	Description	Mean	Std. deviation	Range
Pregnancies	No. of pregnancies	3.85	3.37	0–17
Glucose	2 hours of oral glucose tolerance test for plasma glucose concentration	121	32	0–199
Blood pressure	Blood pressure in mm Hg	69.1	19.3	0–122
Skin thickness	Skinfold thickness of triceps (mm)	20.5	15.9	0–99
Insulin	Two hours of serum insulin (mu U/ml)	79.8	115	0–846
BMI	Body mass index (weight in kg/(height in m)^2^)	32	7.88	0–67
Diabetes Pedigree Function	Attribute used in diabetes prognosis	0.47	0.33	0.078–2.4
Age	Age (years)	33.2	11.8	21–81
Outcome	Class variable (0 or 1)	0.35	0.48	Y/N

**Table 4:** Performance metrics for diabetes classification.

Performance metric	Formula
Recall	TP/(TP+FN)
Precision	TP/(TP+FP)
Accuracy	(TP+TN)/(TP+TN+FP+FN)

**Table 5:** Performance measure for diabetes prediction.

Performance metric	Formula
*r*	$\left(n\left(\sum XY\right)-\left(\sum X\right)\left(\sum Y\right)\right)/\sqrt{\left[n{\sum X}^{2}-{\left(\sum X\right)}^{2}\right]\left[n{\sum Y}^{2}-{\left(\sum Y\right)}^{2}\right]}$
Root mean square error (RMSE)	$\sqrt{\left[\sum_{i=1}^{N}{\left(y_{fi\;}-y_{f0}\right)}^{2}/N\right]}$
Accuracy	(TP+TN)/(TP+TN+FP+FN)

**Table 6:** Forecasting model comparison for BG.

Algorithm	*r*	RMSE	Accuracy
Moving average	0.71	42.946	75.4
Linear regression	−0.071	82.592	72.7
Proposed fine-tuned LSTM	0.999	2.285	87.26

**Table 7:** Proposed prediction method vs. state-of-the-art systems.

Algorithm	Accuracy (%)
J48 [62]	67.9
K-mean [60]	70.5
Feed forward-neural network [63]	71.8
RB-Bayes [64]	72.9
Naive Bayes [65]	76.3
Artificial neural network [61]	85.09
Proposed method (LSTM)	87.26

## Data Availability

The data used to support the findings of this study are included within the article.
